The article "Top-Down Influence Leads to a Reduced Sense of Body Ownership in Individuals With Depersonalization Tendencies: A Focus on Full Body Illusion" was published in 2022. Journal: Front Psychol.

# Top-Down Influence Leads to a Reduced Sense of Body Ownership in Individuals With Depersonalization Tendencies: A Focus on Full Body Illusion

**DOI:** 10.3389/fpsyg.2022.790960

**Published:** 2022-06-02

**Authors:** Kazuki Yamamoto, Takashi Nakao

**Affiliations:** Graduate School of Humanities and Social Sciences, Hiroshima University, Higashihiroshima, Japan

**Keywords:** body ownership, full body illusion, depersonalization, top-down influence, self-association

## Abstract

Sense of body ownership, that is, the feeling that “my body belongs to me,” has been examined by both the rubber hand illusion (RHI) and full body illusion (FBI). In a study that examined the relationship between RHI and depersonalization, a symptom in which people experience a lower sense of body ownership, people with a high depersonalization tendency experienced RHI through the bottom-up process of visual-tactile integration. Why is it that people with depersonalization feel a lower sense of body ownership over their bodies? Case studies of depersonalization suggest that the top-down cognition in people with depersonalization may make them less likely to feel a sense of body ownership. However, the top-down influence on the sense of body ownership in depersonalization has not yet been experimentally demonstrated. By incorporating top-down manipulation (e.g., instructing participants to regard a fake body as their own) into the FBI procedure, we aimed to clarify the cause of the reduced sense of body ownership in people with a high depersonalization tendency. The FBI procedure was conducted in a virtual reality environment using an avatar as a fake body. The avatar was presented from a third-person perspective, and visual-tactile stimuli were presented to create an illusion. To examine the degree of illusion, we measured the skin conductance responses to the fear stimulus presented after the visual-tactile stimuli presentation. The degree of depersonalization was measured using the Japanese version of the Cambridge Depersonalization Scale. To manipulate the top-down influence, we provided self-association instructions before the presentation of the visual-tactile stimuli. We predicted that the higher the degree of depersonalization, the lower the degree of illusion in the self-association instruction. The results showed that participants with a higher depersonalization tendency had a lower degree of illusion (*rho* = −0.424, *p* = 0.035) in the self-association condition. This indicates that in people with a high depersonalization tendency, top-down cognition of the body as their own leads to a decrease in the sense of body ownership.

## Introduction

As we move and observe our bodies, we are confident that our body is our own; this sense is called the sense of body ownership (Gallagher, 2000). Although the sense of body ownership seems to be a consistent feeling, it can be manipulated through specific experimental methods, allowing that sense to be examined and understood. These methods include inducing body illusion phenomena called the rubber hand illusion (RHI) and full body illusion (FBI), which shift the sense of body ownership to objects other than the self-body, such as rubber hands or avatars. In the RHI experiment, the participant’s hand is hidden behind a screen, and only a rubber hand is visible. They are simultaneously touched, giving the participant a sense of body ownership over the rubber hand (Botvinick and Cohen, 1998). In the FBI experiment, the avatar was in front of the participant; both the avatar and the participant’s backs were stroked at the same time, giving the participant the feeling that the avatar was their own body (Nakul et al., 2020). These body illusion experiments indicate that it is possible to shift the sense of body ownership from one’s own body to objects other than one’s own body through bottom-up factors, that is, the spatiotemporal synchronization of visual-tactile information.

In psychopathology, depersonalization is known to show symptoms of body ownership, such as leaving one’s body and lacking a sense of body ownership toward one’s own body. A primary symptom of depersonalization is the experience of feeling unreal or detached, or being an outside observer to one’s own thoughts, feelings, sensations, body, or actions (Sierra, 2009; Sierra and David, 2011; Medford, 2012). Although the DSM-V (American Psychiatric Association, 2013) differentiates between “depersonalization” and “derealization,” as in the name of depersonalization/derealization disorder, these two phenomena often occur concurrently. The depersonalization/derealization disorder distinction may not apply as some patients with persistent depersonalization symptoms experience both phenomena (Sierra, 2009). In this article, as in many studies on the topic, we will use the term “depersonalization” without differentiating between depersonalization and derealization.

Kanayama et al. (2009) examined the RHI in people with a depersonalization tendency and reported results suggesting that people with a high depersonalization tendency can integrate visual-tactile stimuli. They used the Cambridge Depersonalization Scale (CDS; Sierra and Berrios, 2000) to measure healthy participants’ degrees of depersonalization disorder (termed depersonalization/derealization disorder in the DSM-V [American Psychiatric Association, 2013]). Participants were divided into high and low tendency groups based on a cutoff score of 70, which is highly sensitive to patients with depersonalization (Sierra and Berrios, 2000). After the RHI procedure was conducted, a questionnaire measuring the degree of illusion intensity was used to compare the mean of the questionnaire scores (1 = totally disagree, 7 = totally agree) between groups. The results showed that the high tendency group had significantly higher scores on illusion items (e.g., “I felt as if the rubber hand was my hand”) than the low group. This result demonstrates that people with depersonalization can integrate visual-tactile stimuli through a bottom-up process to experience a sense of body ownership.

Top-down influence on the sense of body ownership has been suggested by the RHI study of Tsakiris and Haggard (2005) and the case studies on depersonalization of Hunter et al. (2003). Tsakiris and Haggard (2005) added two conditions to the RHI to make participants recognize that the objects giving the sense of body ownership were not part of their body. In one condition, the rubber hand’s orientation was different from the participant’s hand’s orientation, while in the other condition, a wooden stick was used instead of the rubber hand. After presenting visual-tactile stimuli, the experimenter measured the degree to which the position of the participant’s hands drifted toward the position of the rubber hand (or wooden stick). The results showed no significant difference in RHI in these two conditions. Tsakiris and Haggard (2005) suggest that the sense of body ownership induced by bottom-up integration of visual-tactile stimuli is inhibited by the top-down cognition that a rubber hand with a changed orientation or a wooden stick is not one’s own body. In a review of case studies of depersonalization disorder, Hunter et al. (2003) stated that misattributions of the normally transient symptoms of depersonalization as indicative of severe mental or brain disorders leads to the chronicity of symptoms. In other words, a normally transient experience, such as temporally losing the sense of body ownership, becomes chronic due to a distorted top-down cognition of the experience as serious and an abnormal symptom. Based on previous studies of RHI and depersonalization, it is possible that top-down cognition affects the sense of body ownership, and people with depersonalization tendencies may be less likely to feel a sense of body ownership because of the top-down influence.

However, top-down influence on the sense of body ownership has not yet been verified. Tsakiris and Haggard (2005) manipulated the hand orientation and used a wooden stick, which made it difficult for participants to perceive the correspondence between the stroking position of their own hand and the rubber hand or stick. This may have inhibited the bottom-up visual-tactile integration process, and thus, the observed results cannot be attributed solely to the influence of top-down cognition. In addition, Hunter et al. (2003) derived their claims from case studies, and they needed to be verified. No studies have examined the top-down influence on the sense of body ownership in people with depersonalization.

This study aimed to determine the cause of feeling a lower sense of body ownership in people who have depersonalization tendencies by manipulating the top-down factor (e.g., instructing participants to regard a fake body as if it were their own). In this experiment, we used the FBI paradigm (with the added manipulation of top-down on a fake body) rather than RHI because the main experience of the depersonalized individual involved a full-body sense of body ownership, that is, “feeling as if one were looking at oneself from the outside.” Therefore, we used the FBI paradigm from the third-person perspective (Lenggenhager et al., 2007), in which the object is observed from behind. In this study, we used a virtual reality (VR) environment, and the fake body was an avatar presented in front of participants in the VR.

This study used the illusion questionnaire and the skin conductance response (SCR) as FBI indices. The illusion questionnaire, which is a subjective measure, consists of items related to the FBI, such as “I felt as if the avatar in front of me was my own body” (Lenggenhager et al., 2007; Petkova and Ehrsson, 2008; Salomon et al., 2013). As we instructed participants to regard a fake body as if it was their own, we anticipated that demand characteristics may contaminate subjective ratings. Therefore, the SCR was used as an objective physiological index, and mental sweating was measured electrically when a fear stimulus was presented, such as seeing a fake body being stabbed. The more the participants feel that the fake body is their own body, the larger is the SCR observed (Petkova and Ehrsson, 2008; Guterstam et al., 2015).

To manipulate the top-down factor on the fake body, we applied the manipulation used in the self-prioritization effect study by Sui et al. (2012). In their experiment, participants were instructed to associate geometric shapes (e.g., circles and triangles) with social labels (e.g., self and others). In a subsequent judgment task, they found an effect specific to the self (the reaction time of the judgment was faster and more accurate than those associated with the other). This result shows that their self-association instruction in a top-down manner is an efficient way of constructing associations between objects and the self. In the present experiment, we asked the participants to associate the fake body with the self or another person (e.g., “Look at the avatar’s back while regarding the avatar’s body as your own”) before presenting them with visual-tactile stimuli.

In this study, we included the following three association conditions: non-association condition, in which the FBI paradigm is performed without top-down manipulation; self-association condition, in which the FBI paradigm is performed with the avatar regarded as the self-body by instruction; and the other-association condition, in which the FBI paradigm is performed with the avatar regarded as not the self-body (i.e., another person’s body). The non-association condition was designed to confirm the relationship between RHI and depersonalization (Kanayama et al., 2009) in the FBI. Self-association and other-association conditions were designed to examine the top-down influence. Moreover, in this study, as in other body illusion studies, the degree of illusion was determined by the difference between the synchronous condition (in which the visual-tactile stimuli are presented simultaneously to create the illusion) and the asynchronous condition (in which the presentation of the visual-tactile stimuli is staggered to create less of the illusion). To confirm the relationship between the degree of depersonalization and the amount of FBI induced by visual-tactile integration, we examined the relationship between CDS scores and the degree of illusions in the non-association condition. To examine the relationship between the degree of depersonalization and top-down influence, we examined the correlation between CDS scores and the degree of illusion in the self-association condition in the FBI indices.

The hypotheses of this study are as follows: as in Kanayama et al. (2009), people with a high depersonalization tendency were expected to feel a sense of body ownership over avatars in the absence of top-down manipulation. In other words, it is expected that the higher the degree of depersonalization, the higher the degree of illusion in the non-association condition. However, because of the negative cognition of their own bodies experienced by people with depersonalization (Hunter et al., 2003; Tsakiris and Haggard, 2005), people with a high depersonalization tendency were expected to feel a sense of body ownership over avatars to a lesser degree when they regard the avatar as their own body. In other words, it is expected that the higher the degree of depersonalization, the lower the degree of illusion in the self-association condition.

As a secondary purpose of this study, we investigated the influence of the top-down factor on the FBI. To our knowledge, no study has examined the influence of self-association instruction on the FBI. We examined the effect of self-association instruction on the FBI for people with a low degree of depersonalization. Since we predicted that higher depersonalization scores would lead to a lesser likelihood for the FBI to emerge in the self-association condition, we examined the low depersonalization group.

## Materials and Methods

### Participants

In this experiment, the participants were limited to men, the same sex as the experimenter, because the experimenter was required to stroke the participant’s back. Previous studies have shown that there was no significant difference in the degree of illusions between men and women (Petkova and Ehrsson, 2008; Kilteni et al., 2013); therefore, no gender differences are expected.

As few people have a high degree of depersonalization (American Psychiatric Association, 2013), we screened for depersonalization using the Japanese version of the Cambridge Depersonalization Scale (Tanabe, 2004) when recruiting participants for the experiment. The request for participants was posted on the bulletin board system at Hiroshima University and indicated that male undergraduate and graduate students were eligible.

Of the 157 CDS respondents, those with scores above the cutoff of 70 (Sierra and Berrios, 2000) were considered to have a high degree of depersonalization, whereas those with scores below 70 were considered to have a low degree of depersonalization; individuals from both groups were recruited to participate. Among the respondents, 27 had scores above 70 and 130 had scores below 70. All 27 respondents who scored above 70 points were invited to participate in the experiment, of which only a total of 11 people became participants. In addition, 25 people with scores below 70 were randomly selected and invited to participate in the experiment, and finally, 20 of them became participants. In total, 31 men participated. However, those who did not show a reliable threat-evoked SCR were excluded (four participants, see section Skin Conductance Response below), and the remaining 27 participants were included in the analysis (mean age of 21.26 years, range 18–25 years). The mean CDS score of the 27 participants was 43.65 points, with a range of 10–98 points. Eight participants were above the cutoff of 70 points. Figure 1 shows the number of respondents to the CDS and participants in this experiment in each CDS score group.

**Figure 1:** Number of respondents to the Cambridge Depersonalization Scale (CDS) and participants in this experiment in each CDS score group.

The implementation of the CDS and this experiment was reviewed by the Ethics Review Committee of the Graduate School of Human and Social Sciences, Hiroshima University (approval number 20200100). When recruiting participants, the respondents were informed of the following points prior to completing the questionnaire: (1) An honorarium of 1,000 JPY would be paid for participation in the experiment, which would be conducted on a different day from answering to the questionnaire and (2) not all respondents would be asked to participate in this experiment. They were told to proceed with the questionnaire only if they agreed with the above statements. When conducting the actual experiment, the researcher explained that participation in the experiment was voluntary and that they could stop at any time during the experiment. They were then asked to sign a consent form.

### Depersonalization Questionnaire

The Japanese version of the CDS (Tanabe, 2004) was used to measure the degree of depersonalization. The CDS consists of 29 items reported as depersonalization symptoms, which was a subcategory of dissociative disorders in the DSM-IV at the time (the same applies to the DSM-V). Each item consists of experiences of depersonalization over a six-month period and requires responses on two Likert scales regarding a five-point scale of frequency (0: never–4: always) and a six-point scale of duration (1: few seconds–6: more than a week). However, if the frequency is “0,” then there should be no duration. Therefore, in this study, we added one point (“0: never, and therefore, cannot be answered”) to the scale of duration. The total score of the scale was the sum of the scores of all items (0–290 range). The higher the score, the greater the possibility of depersonalization disorder. Moreover, by setting the cutoff point at 70, the sensitivity for patients with depersonalization has been shown to be 75.5% (Sierra and Berrios, 2000). Examples of items include, “Out of the blue, I feel strange, as if I were not real or as if I were cut off from the world.”

### Equipment

We used a head-mounted display (HMD; Oculus Rift; Display Resolution = 1,200 × 698) to immerse the participants in the VR environment. To synchronize the participant’s head movements with the viewpoint in the VR environment, we used Oculus sensors. The display used for VR was the ProLite G2773HS (Iiyama Inc.).

A skin potentiometer, which was a GSR electrode (Brain Products Inc.), was used to measure the SCR. Brain Amp ExG (Brain Products Inc.) was used to amplify the electrical signals in the physiological indices.

### Stimulation

To induce the illusion, we used a visual stimulus (an animation of a hand stroking up and down 15 cm of the avatar’s back for 90 s) and a tactile stimulus (a stick stroking 15 cm of the participant’s back for 90 s).

To elicit the SCR used to measure the feeling of a sense of body ownership, a fear stimulus (an animation of a knife stabbing the avatar in the back) was presented 90 s after the visual-tactile stimuli were presented.

### Experimental Design

The experiment consisted of two within-participant factors. One was the presentation of the tactile stimulus, which included two conditions: synchronous and asynchronous. The other factor was the instruction for the top-down body association, which included three conditions: non-association, self-association, and other-association. Each participant took part in the experiment under all three top-down body association conditions in both the synchronous and asynchronous conditions.

Regarding the visual-tactile stimuli, the synchronous condition was used to induce the illusion, and the asynchronous condition was not used to induce the illusion. In the synchronous condition, the visual stimulus, the movement of the hand patting the avatar’s back in VR, was synchronized with the tactile stimulus, which was the movement of the stick patting the participant’s back. In the asynchronous condition, when the hand in the VR stroking the avatar moved from top to bottom, the stick stroking the participant’s back moved from bottom to top. Conversely, when the hand in the VR was stroked from bottom to top, the stroking stick stroked the participant’s back from top to bottom.

Regarding the instruction for the top-down body association, after immersing the participants in the VR environment (Figure 2A), the experimenter explicitly gave participants their own labels on the avatar by instruction in the self-association condition. In the other-association condition, the experimenter explicitly gave participants the other-person label on the avatar by instruction. No such instruction for top-down body association was given in the non-association condition, as with the typical FBI procedure. The avatars used in these three conditions differed in brightness (Figure 2B), and the combination of the three conditions and avatar color was randomized among the participants.

**Figure 2:** **(A)** In this experimental environment, we used Unity2018 to create a VR environment that resembles a room, referring to the VR environment used by Slater et al. (2010). The size of the room was 8 m × 6 m, and a male avatar was placed in the center. A VR camera was set up 1.5 m behind the avatar to serve as the viewpoint for the HMD worn by the participants. The height of the VR camera, which is the participant’s point of view in the VR, was adjusted to be the height of the measured participant’s point of view. **(B)** The three colors used were white (R: 255, G: 255, B: 255), gray (R: 127, G: 127, B: 127), and black (R: 0, G: 0, B: 0).

### Indices

#### Illusion Questionnaire

We selected eight items that suited the purpose of this experiment from the FBI questions used by Petkova and Ehrsson (2008) and Romano et al. (2014) to ask about the participants’ experience of the illusion during the 90 s stimulus presentation phase. The questionnaire items were selected based on Gonzalez-Franco and Peck (2018). The content of the questionnaire consisted of two types of items: five illusion items to measure the degree of illusion and three control items to determine participants’ compliance with the FBI task (Table 1). Participants were asked to answer the questionnaire items on a seven-point Likert scale (−3: not at all applicable–3: frequently applicable).

**Table 1:** Items of the illusion questionnaire.

Q1 (Illusion item): It felt like the virtual body was my body
Q2 (Control item): I felt naked
Q3 (Control item): It felt as if my body had turned into a virtual body
Q4 (Control item): I felt as if I had two bodies
Q5 (Illusion item): It seemed as though the touch I felt was caused by the hand touching the virtual body (= I felt tactile sensations from virtual body)
Q6 (Illusion item): I felt as if I was drifting frontwards or backwards
Q7 (Illusion item): It felt like I could control the movement of the virtual body I was looking at
Q8 (Illusion item): I felt like I could not move my own body

#### Skin Conductance Response

The degree of illusion was measured by electrically detecting sweating during the fear stimuli (Petkova and Ehrsson, 2008). The more the avatar is perceived as one’s own body, the greater is the SCR to the knife event (Petkova and Ehrsson, 2008; Guterstam et al., 2015).

### Procedure

#### Pre-experimental Phase

We kept the room temperature constant for all participants to avoid affecting their SCR during the experiment. Specifically, we turned on the air conditioner in the laboratory 1 h before the participants were scheduled to arrive at the laboratory, and adjusted the room temperature to 24°C.

After the participants arrived, we explained the contents of the experiment and showed them how to put on the VR goggles. At that time, we did not tell them about the contents of the illusion. After the explanation, the experimental consent form was explained to the participants.

Following the completion of the consent form, to measure the participant’s skin electricity, the skin potentiometer was attached to the upper first joint of the index and middle fingers of the participant’s left hand. When attaching the potentiometer, the keratin of the skin of the index and middle fingers of the participant’s left hand was removed with SkinPure, a skin pre-treatment gel to reduce skin contact resistance. The remaining SkinPure was wiped off with alcohol-soaked cotton and dry cotton. Then, the skin potentiometer was fixed with tape to prevent detachment during the experiment.

To match the point of view in the VR environment with the participant’s actual point of view, the height of the participant’s point of view was measured with a measuring tape, and the height of the camera’s point of view in the VR environment was adjusted. Then, we told the participants about the size of the HMD, and how to adjust the focus, before asking them to put it on. The participants were then asked to adjust their body orientation so that their point of view was pointed directly at the avatar’s back.

Immersion in a VR environment may cause sickness in people who are not familiar with the VR environment. Therefore, to reduce the possibility of VR sickness during the experiment, we had the participants wear the HMD before the experiment and immerse themselves in the actual experimental environment for 5 min. During this time, the participants were allowed to move their heads freely to get used to the VR environment. After receiving a signal from the participants indicating that they were acclimatized to the VR environment, we moved on to the experimental phase of the FBI.

#### Experimental Phase

All participants started the experiment under the non-association condition because it was expected that the body association would be generated even in the non-association condition if it was conducted after the self-association or other-association conditions. In the non-association condition, participants were asked to put on the HMD at the beginning of the trial, and the synchronous and asynchronous conditions were conducted two times each. The order of the synchronous and asynchronous conditions was randomized for each participant. The participants were instructed to stand and look at the avatar’s back for a 90 s duration of the visual-tactile stimuli. After 90 s of stimulation, a knife appeared and stabbed the avatar’s back (fear stimulus). After the presentation of the fear stimulus, participants were asked to fill out an illusion questionnaire. After completing the questionnaire, we moved on to the next trial.

In the self-association or other-association condition, before presenting the visual-tactile stimuli, the participants were instructed to associate the avatar with self or other (e.g., “Look at the avatar’s back while regarding that the avatar’s body is your own” or “Look at the avatar’s back while regarding that the avatar’s body is a stranger’s body”). The sequence of trials after the instruction was the same as in the non-association condition for both the self-association and other-association conditions.

After completing all the association conditions, the skin electrometer attached to the left hand was removed, and the hand was washed with water to remove the glue residue.

To confirm that the manipulation with the top-down body association instruction was effective, we conducted a matching task for the self-prioritization effect (SPE; Sui et al., 2012). This task was constructed in Psychopy3,^1^ and images (avatars in this study) and social labels (self or other) were presented in each trial. The flow of one trial in the matching task was as follows: In each trial, a gazing point was presented in the center of the screen for 500 ms, and then the avatar-label pairs were presented for 100 ms. The participants were instructed to press the F key if the presented pairs matched the avatar-label pairs they had memorized in the self-association and other-association conditions, and to press the J key if the pairs did not match. If the response key was pressed before 1,500 ms after the presentation of the avatar-label pairs, feedback on whether the answer was “correct” or “incorrect” was presented for 500 ms. If the key press was after 1,500 ms, the feedback “late” was presented (Figure 3). Unlike the typical SPE experiment (Sui et al., 2012), we did not instruct the correspondence between images and social labels before conducting the matching task because they had already been taught during the FBI task. The participants performed 16 trials of a practice task. Following the practice task, the participants moved on to the main task. The main task consisted of three blocks of 48 trials each.

**Figure 3:** Example of one trial series of matching tasks. The flow of one trial in the matching task was as follows. In each trial, a gazing point was presented in the center of the screen for 500 ms, and then the avatar-label pairs were presented for 100 ms. The participants were instructed to press the F key if the presented pairs matched the avatar-label pairs that they had memorized in the self-association condition and other-association condition, and to press the J key if the pairs did not match. If the response key was pressed before 1,500 ms after the presentation of the avatar-label pairs, feedback on whether the answer was “correct” or “incorrect” was presented for 500 ms. If the key press was after 1,500 ms, the feedback “late” was presented.

Finally, after completing the matching task, the participants were asked to fill out forms to receive the honorarium.

### Statistics

As a sampling method, participants were intentionally selected from the high and low CDS score groups. Because of this lack of purely random sampling, the assumption of a normal distribution may have been compromised, and the analysis in this study was conducted using nonparametric tests.

#### Illusion Questionnaire

Initially, for each participant, the mean values of the illusion and control items for each stimulus presentation condition in each association condition were calculated.

After calculating the mean values, a test of the difference between the means (Wilcoxon signed-rank test) of the synchronous and asynchronous conditions was conducted in each association condition to confirm the creation of the illusion. In the non-association condition, a one-tailed test was used because it has been reported that the scores on the questionnaire were higher in the synchronous condition than in the asynchronous condition for the illusion items (Petkova and Ehrsson, 2008; Romano et al., 2014).

To confirm the relationship between the degree of depersonalization and the amount of FBI induced by visual-tactile integration, we examined the relationship between the degree of depersonalization and the degree of illusion in the non-association condition. Kanayama et al. (2009) did not specify whether the questionnaire scores used for comparison were for the synchronous condition or the difference between synchronous and asynchronous scores. In this study, we used the difference between the synchronous and asynchronous conditions as the degree of illusion, in accordance with the degree of illusion commonly used in RHI and FBI studies. Therefore, we used the degree of illusion the difference between the mean values of the illusion item scores for the synchronous and asynchronous conditions in the non-association condition. Then, Spearman’s rank correlation coefficients were calculated between the degree of illusion in the non-association condition and the CDS scores (one-tailed test).

To examine the relationship between the degree of illusion induced by top-down association (self or other) and the degree of depersonalization, the difference between the mean values of the illusion item scores for the synchronous and asynchronous conditions in each association condition was used as the degree of illusion. Then, the Spearman’s rank correlation coefficient between the values calculated as the degree of illusion for each association condition and the CDS scores was calculated.

#### Skin Conductance Response

We extracted the continuous phasic SCR of the obtained skin conductance data by continuous decomposition analysis (CDA) using Ledalab (version 3.2.5^2^; Benedek and Kaernbach, 2010) running in MATLAB 9.7.0 (The Mathworks Inc.). We calculated the phasic SCR (average phasic driver [CDA.SCR]) measured in the 5 s range after the presentation of the fear stimulus. CDA.SCR was calculated for synchronous and asynchronous conditions in each association condition. Referencing Petkova and Ehrsson (2008), participants for whom the SCR elicited by the threats were not reliable (“null responders”), because they had zero response in more than two-thirds of the trials, were excluded from the analysis. As previously stated, four participants did not demonstrate a reliable threat-evoked SCR; thus, their data were excluded from these statistics.

To confirm the creation of illusion, a test of the difference between the average values (Wilcoxon signed-rank test) of the synchronous and asynchronous conditions was conducted for each association condition. In the non-association condition, a one-tailed test was used because it has been reported that the CDA.SCR was higher in the synchronous condition than in the asynchronous condition (Petkova and Ehrsson, 2008).

To confirm the relationship between the degree of depersonalization and the amount of FBI induced by visual-tactile integration, as in the questionnaire, we used as the degree of illusion the difference between the mean values of the CDA.SCR for the synchronous and asynchronous conditions in the non-association condition. Then, Spearman’s rank correlation coefficients were calculated between the degree of illusion in the non-association condition and CDS scores (one-tailed test).

To examine the relationship between the degree of illusion in each association condition and the degree of depersonalization, the difference between the mean values of the CDA.SCR for the synchronous and asynchronous conditions in each association condition was used as the degree of illusion. Then, the Spearman’s rank correlation coefficient between the values calculated as the degree of illusion for each association condition and the CDS scores was calculated.

#### Matching Task

To confirm that the participants could associate avatars of different colors with social labels, we used the Wilcoxon signed-rank test to judge whether the percentage of correct answers for self and other was significantly above the chance level (50%).

In addition, to confirm that the participants were not merely aware of symbolic correspondences between avatars and social labels, but that they associated the avatar with the label “self” with the participant themselves, the occurrence of SPE was also examined. The reaction time and discrimination power (A’) were used to confirm the occurrence of SPE. We classified the trials into Hit (judged to be a match when the pairs match), Miss (judged to be a mismatch when the pairs do not match), Correct Rejection (CR; judged to be a mismatch when the pairs do not match), and False Alarm (FA; judged to be a match when the pairs do not match) trials. The reaction times were calculated as the mean of the correct responses (Hit + CR) trials for each self and other conditions. The Wilcoxon signed-rank test was used to determine whether an SPE occurred when the self-condition was significantly faster than the other conditions. A’ was calculated based on signal detection theory for the self and other conditions, and the Wilcoxon signed-rank test was used to determine whether an SPE occurred when the self-condition was significantly higher than the other conditions.

## Results

### Matching Task

To confirm whether the avatars were associated with the self or the other person by instruction for the top-down body association, we tested the performance of the matching task for the following two points: whether the accuracy was above the chance level and whether SPE occurred.

Regarding accuracy, we examined whether the accuracy for both the self and other conditions was significantly above the chance level (50%). The Wilcoxon signed-rank test showed that both the self and other conditions were significantly above the chance level (Self, *Z* = 4.529, *p* < 0.001, *r* = 0.616, 95% confidence interval [CI] = 0.424, 0.756; Other, *Z* = 3.904, *p* < 0.001, *r* = 0.531, 95% CI = 0.314, 0.696; Figure 4A).

**Figure 4:** **(A)** Mean values of accuracy for self and other conditions. **(B)** Mean values of reaction time for the correct response trials of the self and other conditions. **(C)** Mean values of A’ for the correct response trials of each condition (***p < 0.001, error bars are SEs).

For SPE, we calculated A’ and the mean reaction time for the correct response trials of the self and other conditions. The Wilcoxon signed-rank test was used to examine the differences between the self and other conditions for these indices. The results showed that the self-condition had a significantly shorter reaction time than the other condition (*Z* = −3.976, *p* < 0.001, *r* = −0.541, 95% CI = −0.703, −0.327; Figure 4B), and that the self-condition had a significantly higher A’ than the other condition (*Z* = 3.962, *p* < 0.001, *r* = 0.539, 95% CI = 0.324, 0.701; Figure 4C).

These results confirmed that the manipulation with the top-down body association instruction was effective.

### Checking for Inappropriate Responses to the Illusion Questionnaire

First, to examine whether the participants gave incorrect answers to the illusion questionnaire (e.g., answering without reading the item content), we tested whether no significant difference was found between the synchronous and asynchronous conditions in the control items, unlike in the case of the illusion items. The Wilcoxon signed-rank test showed that there was no significant difference between the synchronous and asynchronous conditions in all the top-down body association conditions (non-association, *Z* = 1.614, *p* = 0.106, *r* = 0.220, 95% CI = −0.043, 0.454; self-association, *Z* = 1.778, *p* = 0.075, *r* = 0.242, 95% CI = −0.020, 0.473; other-association, *Z* = 1.339, *p* = 0.162, *r* = 0.190, 95% CI = −0.074, 0.430; Figure 5A).

**Figure 5:** **(A)** Mean scores of control items for the synchronous and asynchronous conditions for each top-down body association condition. **(B)** Mean scores of illusion items for synchronous and asynchronous conditions for each top-down body association condition. **(C)** Mean CDA.SCR for the synchronous and asynchronous conditions for each top-down body association condition (***p < 0.001, **p < 0.01, error bars are SEs).

### Confirmation of the Full Body Illusion Creation for All Participants

To confirm the creation of the FBI, the mean scores of the illusion items were calculated for each combination of visual-tactile stimuli conditions and the top-down body association conditions in the illusion questionnaire and CDA.SCR. Comparison of the difference in the mean values between the synchronous and asynchronous conditions was conducted for each of the top-down body association conditions.

In the illusion questionnaire, the Wilcoxon signed-rank test showed that there were significant differences between the synchronous and asynchronous conditions in the non-association and self-association conditions (non-association, *Z* = 4.036, *p* < 0.001, *r* = 0.549, 95% CI = 0.337, 0.708, one-sided test with lower boundary; self-association, *Z* = 3.579, *p* < 0.001, *r* = 0.487, 95% CI = 0.259, 0.663; Figure 5B), and no significant difference was found in the other-association condition (*Z* = 1.800, *p* = 0.072, *r* = 0.245, 95% CI = −0.017, 0.475; Figure 5B). In the non-association and self-association conditions, the scores were higher in the synchronous condition than in the asynchronous condition. Thus, the FBI was confirmed to have been created under those two conditions in the illusion questionnaire.

In the SCR, the Wilcoxon signed-rank test showed that there were significant differences between the synchronous and asynchronous conditions only in the self-association condition (*Z* = 3.111, *p* = 0.002, *r* = 0.423, 95% CI = 0.183, 0.616; Figure 5C), and no significant difference was found in the non-association and other-association conditions (non-association, *Z* = 1.357, *p* = 0.087, *r* = 0.185, 95% CI = −0.080, 0.425, one-sided test with lower boundary; other-association, *Z* = −1.910, *p* = 0.056, *r* = −0.260, 95% CI = −0.487, 0.001; Figure 5C). Thus, only the self-association condition was confirmed to have created the FBI in the SCR.

### Relationship Between the Degree of Depersonalization and Amount of FBI Induced by Visual-Tactile Integration

Similar to Kanayama et al. (2009), by analyzing the data in the non-instruction condition, we investigated the relationship between the degree of depersonalization and the amount of FBI induced by visual-tactile integration. Kanayama et al. (2009) showed that the high tendency group had significantly higher scores on illusion items (e.g., “I felt as if the rubber hand was my hand”) than the low group in the RHI (however, it was not specified whether the scores obtained were for the synchronous condition or for the difference between synchronous and asynchronous conditions). As Kanayama et al. (2009) did not provide any association for the top-down body association, we used the present experiment’s data in the non-association condition. Therefore, we examined the relationship between the CDS score and the degree of FBI (the difference in the value of each index between the synchronous and asynchronous conditions) in the non-association condition. In the illusion questionnaire, we calculated Spearman rank correlation coefficients with age as a control variable. In contrast to the results of Kanayama et al. (2009), there was no significant correlation (*rho* = 0.193, *p* = 0.172, one-sided test with lower boundary; Table 2). Figure 6A shows a scatter plot of the ranks of the illusion questionnaire scores and CDS scores, with age as a control variable.

**Table 2:** Spearman’s rank correlation coefficients between the Cambridge Depersonalization Scale (CDS) scores and degree of full body illusion (FBI; the difference in the value of each index between the synchronous and asynchronous conditions) in each top-down body association condition.

		Illusion questionnaire			SCR		
		Non	Self	Other	Non	Self	Other
CDS scores	*rho*	0.193	0.121	−0.059	0.081	−0.424^*^	0.070
	95% CI	−0.210, 0.540	−0.280, 0.485	−0.436, 0.336	−0.325, 0.461	−0.701, −0.034	−0.334, 0.453

* *p < 0.05*.

*In the illusion questionnaire, the control variable is age. In the SCR, the control variable is age and the overall mean of the non-association condition*.

**Figure 6:** Each scatter plot shows the ranked data. The solid line denotes a regression line. **(A)** Scatter plots for the CDS scores and the value of difference in the illusion items’ scores between the synchronous condition and asynchronous condition in the non-association condition with the age controlled. **(B)** Scatter plots for the CDS scores and the value of difference in CDA.SCR between the synchronous condition and asynchronous condition in the non-association condition with the age and the overall mean of the non-association condition as control variables. **(C)** Scatter plots for the CDS scores and the value of difference in the illusion items’ scores between the synchronous condition and asynchronous condition in the self-association condition with the age controlled. **(D)** Scatter plots for the CDS scores and the value of difference in the illusion items’ scores between the synchronous condition and asynchronous condition in the other-association condition with the age controlled. **(E)** Scatter plots for the CDS scores and the value of difference in CDA.SCR between the synchronous condition and asynchronous condition in the self-association condition with the age and the overall mean of the non-association condition as control variables. **(F)** Scatter plots for the CDS scores and the value of difference in CDA.SCR between the synchronous condition and asynchronous condition in the other-association condition with the age and the overall mean of the non-association condition as control variables.

However, individual differences in SCR amplitude may reflect individual differences in depersonalization independent of the amount of FBI. This possibility was suggested by previous studies on emotional responses to depersonalization; Michal et al. (2013) showed that people with a high degree of depersonalization have a high SCR amplitude in response to sound stimuli. Moreover, a review by Horn et al. (2020) suggested that people with depersonalization produced higher SCR amplitudes because the increased arousal caused by the abnormally high sympathetic arousal of people with depersonalization. Actually, the SCR of both the synchronous and asynchronous conditions in the non-association condition was positively correlated with the degree of depersonalization (synchronous condition, *rho* = 0.552, *p* = 0.003, one-sided test with lower boundary; asynchronous condition, *rho* = 0.338, *p* = 0.091). As individuals with a larger SCR can show a larger SCR difference between two conditions (e.g., synchronous and asynchronous conditions), regardless of the degree of FBI, we used the average of the SCR values for the synchronous and asynchronous conditions in the non-association condition as a control variable to examine the relationship between depersonalization and FBI. Henceforth, we refer to this control value as the SCR control variable.

We calculated Spearman’s rank correlation coefficients between the CDS score and the degree of FBI in SCR (the difference in the value of each index between the synchronous and asynchronous conditions) with the controlling age and SCR control variable. The results of this analysis showed that there was no significant correlation (*rho* = 0.081, *p* = 0.351, one-sided test with lower boundary; Table 2). Figure 6B shows a scatter plot of the ranks of the CDA.SCR and CDS scores, with age and the overall mean of the non-association condition as control variables.

### Examination for the Main Purpose: The Relationship Between the Degree of Depersonalization and the Degree of Illusions in the Association Conditions

We examined the relationship between the CDS score and the degree of FBI (the difference in the value of each index between the synchronous and asynchronous conditions). In the illusion questionnaire, we calculated the Spearman rank correlation coefficients with age as a control variable. The results showed there were no significant correlations (self-association, *rho* = 0.121, *p* = 0.557, 95% CI = −0.280, 0.485; other-association, *rho* = −0.059, *p* = 0.776, 95% CI = −0.436, 0.336; Table 2). Figures 6C,D show a scatter plot of the ranks of the CDS scores and the illusion questionnaire scores in the association conditions, with age as a control variable.

In the SCR, we calculated Spearman’s rank correlation coefficients between the CDS scores and the degree of FBI (the difference between the mean values of the CDA.SCR for the synchronous and asynchronous conditions) in the self- or other-association condition. In these correlation analyses, age and the SCR control variable were included as control variables as there were significant correlations between SCR difference (synchronous–asynchronous) and the SCR control variable both in the self- and other-association conditions (self-association, *rho* = 0.496, *p* = 0.009, 95% CI = 0.143, 0.737; other-association, *rho* = −0.515, *p* = 0.006, 95% CI = −0.749, −0.168). The results showed that there was a significant negative correlation in the self-association condition (*rho* = −0.424, *p* = 0.035, 95% CI = −0.701, −0.034; Table 2), and no significant correlations were found in the other-association condition (other-association, *rho* = 0.070, *p* = 0.740, 95% CI = −0.334, 0.453; Table 2). Figures 6E,F show a scatter plot of the ranks of the CDS scores and the CDA.SCR in the association conditions, with age and the overall mean of the non-association condition as control variables.

### Subsidiary Purpose: Examining the Influence of Top-Down Factors in the FBI

To examine the top-down influence on the FBI, we examined the creation of illusion in 19 participants with a low depersonalization tendency (CDS scores below 70). The degree of illusion (the difference in the value of each index between the synchronous and asynchronous conditions) was compared between the self-association and other-association conditions. In the illusion questionnaire, we compared the mean values of the illusion item scores between the self-association and other-association conditions, and the Wilcoxon signed-rank test showed significant differences between the self-association and other-association conditions (*W* = 121, *p* = 0.037, *r* = 0.582, 95% CI = 0.123, 0.836; Figure 7A). With the SCR, we compared the mean values of CDA.SCR between the self-association and other-association conditions. The Wilcoxon signed-rank test showed a significant difference (*W* = 154, *p* = 0.016, *r* = 0.621, 95% CI = 0.211, 0.845; Figure 7B). In both the illusion questionnaire and the SCR, the FBI was created more in the self-association than in the other-association conditions.

**Figure 7:** Results for participants with a low degree of depersonalization (*p < 0.05, error bars are SEs). **(A)** The value of difference in the illusion items’ scores between the synchronous condition and asynchronous condition in the self-association and other-association conditions for participants with a low degree of depersonalization. **(B)** The value of difference in CDA.SCR between the synchronous condition and asynchronous condition in the self-association and other-association conditions for participants with a low degree of depersonalization.

## Discussion

### Relationship Between Depersonalization and Sense of Body Ownership

This study aimed to clarify that the top-down factor (e.g., instructing people to regard a fake body as their own) causes a lower sense of body ownership in people with depersonalization tendencies. Consistent with the study’s hypothesis, a significant negative correlation between the CDS scores and degree of illusion in the self-association condition was found in the SCR (Figure 6D). This result demonstrated, for the first time, that people with depersonalization have a reduced sense of body ownership when they regard the body as their own in a top-down manner. In other words, people who feel a lower sense of ownership of their own body tend to find it difficult to feel a sense of ownership over an avatar that is regarded as one’s own body in top-down manner.

The top-down process of depersonalization behind the present result remains unknown. The negative cognition of the individuals with depersonalization tendencies for their bodies is one of the factors that contribute to the top-down process. As Hunter et al. (2003) summarized, people with depersonalization have a negative and distorted cognition of their own symptoms. The negative cognition about their own body would arise, which brings about such unwanted symptoms. This negative cognition may be applied to avatars by regarding avatars as their bodies in a top-down manner, which inhibited the FBI. Although we did not measure the negative cognition about their own body and avatar, future studies are needed to determine whether they have a negative cognition of their own body and self-associated avatar.

Another hypothesis, that the higher the degree of depersonalization, the higher the degree of illusion in the non-association condition, was not supported (Figures 6A,B). However, as no negative correlation was observed, there was also no evidence that a sense of ownership through visual-tactile integration was impaired in depersonalization. Besides, the FBI was observed across participants, including those with depersonalization tendencies in the non-association condition (Figure 5B). Taken together with the fact that Kanayama et al. (2009) reported that RHI occurred more in depersonalization, bottom-up visual-tactile integration is likely to be maintained in people with depersonalization tendencies.

One possible reason why a positive correlation similar to the one reported by Kanayama et al. (2009) was not found in this study was that the difference in the target area of the sense of body ownership was manipulated. Both the RHI and the FBI agree that they manipulate the sense of body ownership by presenting visual-tactile stimuli simultaneously; however, they differ in that the sense of body ownership manipulated is either a part of the body or the whole body. The differences between body parts and the whole body have been examined, and neuroimaging studies examining their visual representation have shown that information about body parts and the whole body are represented in separate neural bases (Taylor et al., 2007; Brandman and Yovel, 2016). The RHI and FBI also differ in terms of the onset time of the illusions: in the RHI, the onset time is less than 15 s (Lloyd, 2007), whereas in the FBI, the onset time is 28 s—a difference of about 10 s (O’Kane and Ehrsson, 2021). Although the reason for this difference has not yet been clearly examined, it is possible that the larger the target of the manipulated sense of body ownership, the longer it takes for the illusion to be generated. Based on these findings, it is suggested that the discrepancy between the results of the study of Kanayama et al. (2009) on RHI and the results of the present study on the FBI may be due to the difference in the target of the sense of body ownership being manipulated.

The present findings are based on the results of the SCR in the illusion questionnaire, as there was no significant correlation between the CDS score and the degree of illusion in the self-association condition (Figure 6C). There was also no significant correlation between the CDS scores and the degree of illusion in the non-association condition (Figure 6A). The lack of a significant correlation in the illusion questionnaire may be due to the influence of required characteristics on the answers to the illusion questionnaire. Hunter et al. (2003) stated that people with depersonalization disorders fear being identified as different from others because of their sense of depersonalization. In light of our findings, it is possible that participants with a high depersonalization tendency stated that they felt a sense of body ownership even though they did not experience it in the self-association condition. Thus, it is possible that in the non-association condition, the participants answered that they did not feel a sense of body ownership, even though they felt a strong sense of body ownership toward the avatar. However, it is unclear how the participants cognized the avatar, and hence, it is necessary to test this possibility in a future study. As the SCR is less likely to reflect the subjective bias of the participants, the above possibilities were avoided.

### Examining the Influence of Top-Down Factors in the FBI

Based on the cutoff point in Sierra and Berrios (2000), we examined how top-down factors, such as self-association, influence the degree of illusion in participants with a low and high depersonalization tendency. The reason for examining the participants separately was that we expected that the degree of illusion in the self-association condition would differ between participants with low and high depersonalization tendencies, and the higher the degree of depersonalization, the lower the degree of illusion (Figure 6E). In participants with a low depersonalization tendency, the FBI was observed in the self-association condition rather than the other-association condition on the illusion questionnaire and the SCR (Figures 7A,B). This result demonstrates, for the first time, the influence of top-down factors on the sense of body ownership, as suggested by the previous studies (Tsakiris and Haggard, 2005; Aspell et al., 2009), by manipulating the top-down influence on the fake body.

This result indicates that we should be careful not to form a top-down influence of the fake body, even in typical procedures of body illusion experiments. For example, participants may notice that the experimenter is trying to cognize a fake body as their own body through repeated measurement of the illusion questionnaire and will intentionally or unintentionally try to cognize that as their own body in a top-down manner. In this case, the observed illusion can be contaminated by factors other than visual-tactile stimuli integration or top-down influence. In future research, it will be necessary to conduct experiments and interpret the results by considering the effects of the formation of such a top-down influence.

### Matching Task

We conducted the matching task to check whether the participants could associate an avatar with the self by the self-association instruction (e.g., “Look at the avatar’s back while considering that the avatar’s body is your own”). The results of reaction time and A’ were similar to those of Sui et al. (2012), indicating that self-association manipulation by association with the avatar was properly performed. Considering that the influence of top-down on the FBI was also observed (Figures 7A,B), the manipulation of association introduced in this study is considered to be effective as a manipulation of top-down influence for body ownership. The self-association instruction introduced in this study would be useful for manipulating top-down influence on the body in future research.

### Limitations

The following three limitations of this study should be noted. First, in the non-association condition, the difference in the SCR between the synchronous and asynchronous conditions, predicted based on previous studies (Lenggenhager et al., 2007; Petkova and Ehrsson, 2008), was not observed in this study (Figure 5C). This result might be observed because the SCR in the non-association condition was contaminated by the effect of the surprise caused by observing the fear stimulus for the first time after the illusion induction. The non-association condition was performed first to avoid forming the top-down influence in the non-association condition by conducting it after the self-association and other-association conditions. In the non-association condition, the order of presentation was randomized across participants. As a result, in the synchronous or asynchronous conditions in the initially conducted non-association condition, a large SCR might be evoked due to surprise, making it difficult to observe the differences between the synchronous and asynchronous conditions on average across participants. To avoid as much surprise as possible in future studies, it will be necessary to present the fear stimuli in several practice trials before conducting the experimental conditions.

Second, the process behind the present results, in which the participant with a higher depersonalization tendency showed less FBI when the avatar was self-associated in a top-down manner (Figure 6D), remains unclear. Although the negative body cognition in depersonalized people is thought to explain the present results in the self-association condition, whether the participants with a high depersonalization tendency had negative body cognition was not examined. Collecting the participants’ subjective reports will be necessary to confirm whether depersonalized people negatively cognized the fake body. Even if they negatively cognize the avatar, it is expected that obtaining the actual participant’s cognition in the subjective report will be difficult, as people with depersonalization are often fearful of their own dissimilarity to others and deny their circumstances (Hunter et al., 2003). Thus, it would be useful to measure negative body cognition using cognitive tasks, such as the affective priming paradigm (Fazio et al., 1986) and implicit association test (Greenwald et al., 1998).

Finally, this study did not include people diagnosed with depersonalization. To generalize the present findings to clinical populations, it is necessary to conduct a similar study with a clinical group.

### Conclusion

The results of this study suggest that while people with depersonalization can feel body ownership by integrating visual-tactile stimuli, they are less likely to feel a sense of body ownership when they cognize themselves in their own bodies. These findings may lead to the improvement of symptoms, such as difficulty in feeling body ownership, in people with depersonalization. If people with depersonalization can feel a sense of body ownership by integrating visual-tactile stimuli, then creating a state in which they can visually confirm that they are touching their own body when they feel depersonalization may give them a sense of body ownership. In addition, it was suggested that top-down cognition makes it difficult to feel body ownership, and an approach that improves top-down cognition is important for the treatment for depersonalization.

## Data Availability Statement

The raw data supporting the conclusions of this article will be made available by the authors, without undue reservation.

## Ethics Statement

The studies involving human participants were reviewed and approved by the Ethics Review Committee of the Graduate School of Human and Social Sciences, Hiroshima University. The patients/participants provided their written informed consent to participate in this study.

## Author Contributions

KY and TN contributed to the design of the study and revision of the manuscript. KY conducted the study, analyzed the data, and wrote the first draft. All authors contributed to the article and approved the submitted version.

## Funding

This research was supported by the Center of Innovation Program of the Japan Science and Technology Agency (JST) JPMJCE1311, JPMJCA2208, and by J0A2001.

## Conflict of Interest

The authors declare that the research was conducted in the absence of any commercial or financial relationships that could be construed as a potential conflict of interest.

## Publisher’s Note

All claims expressed in this article are solely those of the authors and do not necessarily represent those of their affiliated organizations, or those of the publisher, the editors and the reviewers. Any product that may be evaluated in this article, or claim that may be made by its manufacturer, is not guaranteed or endorsed by the publisher.

## Footnotes

^1^ https://www.psychopy.org/

^2^ http://www.ledalab.de/documentation.htm
